The article "Comparative Analysis of Early Clinical Features and Complications of Different Types of Acute Pancreatitis" was retracted in 2023. Reasons: suspected computer-generated content; unreliable results or conclusions; concerns about the data; concerns about the results or conclusions.

# Comparative Analysis of Early Clinical Features and Complications of Different Types of Acute Pancreatitis

**DOI:** 10.1155/2022/3771610

**Published:** 2022-06-25

**Authors:** Hongsheng Wu, Keqiang Ma, Biling Liao, Tengfei Ji, Shengmin Zhang, Tiansheng Cao

**Affiliations:** Department of Hepatobiliary Pancreatic Surgery, Affiliated Huadu Hospital, Southern Medical University, Guangzhou, 510800 Guangdong Province, China

## Abstract

**Background:**

Acute pancreatitis (AP) is a common surgical acute abdomen. Different kinds of pancreatitis may have different pathophysiological characteristics each other. The objective of this research was to investigate the early clinical features and complications of different types of acute pancreatitis.

**Methods:**

787 AP patients admitted in the Huadu District People's Hospital of Guangzhou during January 2009 and December 2019 were analyzed retrospectively. Among 787 AP patients, 520 (66.1%) were biliary AP (group I), 69 (8.7%) were alcoholic AP (group II), and 198 (25.2%) were hypertriglyceridemic AP (group III). According to the local and systemic complications and mortality in the early stage, we compared and analyzed the clinical characteristics and prognosis of different types of pancreatitis.

**Results:**

Mild acute pancreatitis accounted for the highest proportion (79.4%) in group I, while moderately severe acute pancreatitis in group II (36.2%) and severe acute pancreatitis in group III (62.6%). In terms of severity score of the pancreatitis, the average scores of BISAP, Ranson, APACHE-II, and MCTSI of the patients in group III were the highest (*p* < 0.01). The incidence of acute peripancreatic fluid collection and infectious pancreatic necrosis was the highest in group III. The incidences of acute necrotic collection, pancreatic pseudocyst, and walled-off necrosis in group III were significantly higher than those in the other two groups (*p* < 0.01). The incidences of systemic inflammatory response syndrome, sepsis, multiple organ failure, intra-abdominal hypertension, and mortality were highest in group III.

**Conclusions:**

There is an upward trend of the incidence rate of hypertriglyceridemic AP in recent years; it has been gradually developed into the second type of acute pancreatitis which is second only to the acute biliary pancreatitis. It is worthy to pay more and more attentions to it due to the feature of its younger onset, high incidence of complications, and high mortality.

## 1. Introduction

Acute pancreatitis (AP) is caused by abnormal activation of digestive enzymes from pancreas which lead to self-digestion of pancreas and peripancreatic organs under various pathogenic factors. Although the etiology of AP is various and complicated, however, among all of these etiologies, biliary stones, alcoholism, and hyperlipidemia are the three main causes which lead to AP. Based on the etiology of AP, acute biliary pancreatitis and alcoholic pancreatitis are the two major causes of acute pancreatitis from the developed countries at present, and two types of these acute pancreatitis accounts for about 80% of the incidence rate of acute pancreatitis [1]. In China, these two kinds of pancreatitis were the most common clinical types of AP in the past. However, in recent years, with the improvement of people's living quality and the changes of diet styles increasingly, the incidence rate of hypertriglyceridemia caused by lipid metabolism disorders has been increasing year by year, which makes the acute pancreatitis caused by hypertriglyceridemia rapidly increase in recent years, and had become one of the common causes of AP [2–5]. The characteristics of its rapid and serious illness, its poor prognosis, and its high mortality rate had attracted the attention of clinicians. Although self-digestion of pancreas and peripancreatic tissue by abnormal activation of pancreatic digestive enzymes is the common feature of acute pancreatitis, however, due to the diversity of etiology of AP, pathophysiological characteristics of acute pancreatitis caused by different etiology may be different [6, 7]. Therefore, it is still unclear whether the diversity of AP etiology affects the incidence of complications in early stage or influenced severity of illness or determines the prognosis. Therefore, the motivation of our study is to explore the relationships between the characteristics of acute pancreatitis and the clinical types of AP and provide theoretical basis for the treatment and prevention of clinical pancreatitis. Thus, we analyzed the data of the AP patients which were admitted in a single medical center during the past 10 years retrospectively and reported.

## 2. Materials and Methods

### 2.1. Materials

787 AP patients admitted to the Guangzhou Huadu District People's Hospital from 2008 to 2018 were enrolled in this research, and all the patients were hospitalized with acute abdominal pain as the main clinical symptom. After admission, they had been made a diagnosis of AP according to the following characteristics (meets all three): (1) abdominal pain; (2) serum amylase level was more than three times higher than the upper limit of normal value; (3) abdominal CT examination showed that the pancreas was swollen with varying degree. From all of the patients, there were 376 males and 411 females with a sex ratio of 1 : 1.09 and an average age of 49.7 ± 3.2 years. Among them, 520 cases (66.1%) were acute biliary AP (group I), 69 (8.7%) were alcoholic AP (group II), and 198 (25.2%) were hypertriglyceridemic AP (group III). According to different types of AP, diagnostic criteria of acute biliary pancreatitis [8], with clinical manifestations of AP, B-ultrasound, CT or MRCP imaging, or endoscopy showed biliary stones. The diagnostic criteria of alcohol-related pancreatitis [9] were as follows: patients with AP clinical symptoms and signs, alcoholic pancreatitis generally requires drinking more than eight alcoholic drinks/day (>100 g/d) for more than 5 years, or drinking alcohol one week before onset of the disease and excluding other etiologies which lead to AP. The diagnostic criteria of hypertriglyceridemic AP are as follows [10]: patients with AP clinical symptoms and signs and the serum triglyceride≥1000 mg/dL in the acute setting. Exclusion criteria are as follows: other types of etiologies which lead to AP, any severe systemic illness, and those with incomplete case files. The basic clinical data of this study is shown in Table 1. This study was approved by the ethics committee of our hospital; due to this was a retrospective study, our ethics committee granted an authorisation to waive written informed consent from patients.

### 2.2. Methods

#### 2.2.1. Patients

According to the classifications from the latest Chinese guidelines for the diagnosis and treatment of acute pancreatitis [11], patients with AP were divided into three groups: acute biliary AP (group I), alcoholic AP (group II), and hypertriglyceridemic AP (group III). The clinical characteristics, clinical classification, bedside index for severity in acute pancreatitis (BISAP) score [12], APACHE-II score [13], Ranson score [14] for severity assessment, modified CT severity index (MCTSI) score [15], and early local and systemic complications were statistically analyzed from each group. Multiple scoring systems were used to evaluate the severity and prognosis of AP. The early local complications included the following: (1) acute peripancreatic fluid collection (APFC) [16]: CT scan imaging feature indicated fluid accumulation with uniform signal and lack of intact capsule in the space of intrapancreatic or peripancreatic tissue; (2) acute necrotic collection (ANC) [17]: ultrasound or MRI indicated necrotic tissue contains in the liquid collection; (3) pancreatic pseudocyst (PPC) [18]: ultrasonography, CT scan, or MRI manifestation showed pancreatic cystic mass, containing pancreatic secretion, granulation tissue, and fibrous tissue; (4) walled-off necrosis (WON) [19]; and (5) infected pancreatic necrosis (IPN) [20]: the indication of the CT scan had typical “bubble sign” around the pancreas. Early systemic complications included the following: (1) systemic inflammatory response syndrome (SIRS) [21], (2) organ failure (OF); and (3) sepsis.

### 2.3. Statistical Analysis

SPSS 12.0 medical statistical software (SPSS, Inc., Chicago, IL, USA) was used for data statistics, continuous data were tested for normal distribution and were expressed in mean differences ± standard deviation ($\bar{x}\pm s$), and *t*-test was used for comparison; the comparison of dichotomous data was presented as *n* (%), and chi-square test was performed for comparison. When comparison involved beyond two groups, Cuzick trend chi-square test (multiple groups) was used. For all the statistical tests, a 0.05 significance level was used to claim a statistically significant effect.

## 3. Results

### 3.1. Clinical Type of AP between Three Groups

Among 520 AP patients in group I, there were 413 cases (79.4%) of MAP, 75 cases (14.4%) of MSAP, and 32 cases (6.2%) of SAP; among 69 AP patients in group II, there were 21 cases (30.4%) of MAP, 25 cases (36.2%) of MSAP, and 23 cases (33.4%) of SAP; for group III, there were 21 cases (10.6%) of MAP, 53 cases (26.8%) of MSAP, and 124 (62.6%) cases of SAP. The ratios of MAP from group I, group II, and group III were 79.4%, 30.4%, and 10.6%, respectively, and there had the difference between the three groups which was statistically significant (*p* < 0.01). The results of clinical classification between the three groups are shown in Table 2.

### 3.2. Severity Scores of Different Types of AP between Three Groups

The average BISAP scores of AP patients from group I, group II, and group III were 2.1 ± 0.8, 2.4 ± 1.3, and 4.5 ± 1.2, respectively; the average BISAP score of group III was significantly higher than that in group I and group II (*p* < 0.01); average Ranson score of three groups were 2.5 ± 0.3, 2.8 ± 0.1, and 5.9 ± 0.4, respectively; average Ranson score of group III was significantly higher than that in group I and group II (*p* < 0.01); the average APACHE-II score of three groups were 8.4 ± 1.6, 15.2 ± 2.3, and 20.12 ± 3.1, respectively; AP patients from the group III had the significantly higher APACHE-II score than that from the other groups (*p* < 0.01); the average MCTSI scores of the three groups were 3.5 ± 0.8, 6.4 ± 1.1, and 9.2 ± 1.3, respectively; similarly, AP patients from the group III had the significantly higher MCTSI score than that from the other groups, and the difference was statistically significant (*p* < 0.01). The results of severity scores of three groups are shown in Table 2; the comparison of clinical classification and severity score between three groups was shown in Figures 1 and 2.

### 3.3. Comparison of Early Local and Systemic Complications among the Three Groups

From the comparison of local complications in early stage, among these complications, APFC complicated in group I, group II, and group III was 17.1%, 65.2%, and 88.9%; ANC complicated in three groups were 12.5%, 11.6%, and 66.7%; PPC complicated in three groups were 4.0%, 4.3%, and 44.9%; WON complicated in three groups were 1.5%, 2.9%, and 39.4%; IPN complicated in three groups were 0.4%, 2.9%, and 32.8%, respectively. The trend chi-square test result indicated that the difference of incidence of APFC, WON, and IPN was statistically significant between three groups each other (*p* < 0.01); for ANC and PPC, incidences occurred in group III were significantly higher than in group I or group II (*p* < 0.01). The incidences of systemic complications in early stage of AP from groups I, II, and III were (40.8% vs. 39.1% vs. 94.4%), organ failure (3.1% vs. 7.2% vs. 88.4%), sepsis (0.4% vs. 2.9% vs. 6.1%), intraperitoneal hypertension (1.3% vs. 50.7% vs. 85.4%), and mortality (0.4% vs. 1.4% vs. 4.0%); comparisons indicated incidences of early systemic complications and mortality were statistically significant between three groups each other (*p* < 0.01). The comparison of the results of early local and systemic complication mortality among the three groups is shown in Figures 3 and 4.

## 4. Discussion

Since updated through the Pancreatic Branch Committee of Chinese Medical Association from 2013, the guidance about AP diagnosis and treatment had been improved obviously, and the rationalization and standardization of the treatment for acute pancreatitis significantly reduced the mortality rate in China. However, as a common surgical acute abdomen, the mortality rate of MSAP and SAP is still about 5.9% [11]. The irrecoverable organ function and uncontrollable infection are the main factors which cause death [22–25]; meanwhile, local and systemic complications caused by acute pancreatitis prolong the hospitalization time and increase the medical expenses [26, 27]; especially for SAP, the incidence of local complications was as high as 59% [28] and has the highest mortality among all types of AP. Therefore, under this situation, clinical surgeons should pay more and more attentions of illness assessment in early stage, organ function protection, infections control, and complications prevention of patients with acute pancreatitis.

The pathogenesis of ABP is due to the obstruction of the common bile or pancreatic duct by the stones from biliary system, which leads to the increase of pancreatic duct pressure, thereby result in activation of pancreatic digestive enzymes [29, 30]. Due to most of the bile duct stones can be proved from the patient's history or hospital auxiliary examination such as B-ultrasound, CT, or MR, therefore, ABP has the definite etiology and early surgery or endoscopic ERCP removal of stones from the bile-pancreatic duct can achieve the purpose of treatment [31–33], and the endocrine and exocrine functions of pancreas were not significantly affected in most mild or moderate AP patients after the etiology was removed [34]. From the research of complications and prognosis of severe BAP, the result of Barauskas et al. [35] indicated that although there was no significant difference about severity scoring between acute biliary AP and alcoholic AP, however, the incidence of complications such as intra-abdominal hypertension (IAH), abdominal compartment syndrome (ACS), and pancreatic necrosis was significantly lower in acute biliary AP than in alcoholic AP, and the mortality was significantly lower than that in alcoholic AP.

Alcoholic AP defined as damage of pancreatic cytotoxic action from the alcohol and its metabolites from the long-term large-scale alcohol intake [36, 37], due to the long-term and high alcohol consumption, most of this kind of patients complicate with chronic pancreatitis or pancreatic fibrosis [38, 39] and even involve other organs such as alcoholic liver damage [40] or chronic renal damage [41]. Therefore, once acute alcoholic pancreatitis occurs, local or systemic complications are more likely to arise from other organs damage aggravation and even lead to multiple organ failure. Several clinical studies [42, 43] have shown that compared with ABP, alcoholic AP, alcoholic AP had higher incidence of complications and poor prognosis. From this study, the results indicated that incidences of local complications in early stage such as APFC, WON, and IPN were significantly higher in alcoholic AP than those in ABP; similarly, systemic incidences of complications of MODS, SIRS, and sepsis were higher in alcoholic AP, and the difference was statistically significant. It was proved the proposition that compared with ABP, alcoholic pancreatitis had the worse illness and poor prognosis.

Hypertriglyceridemic pancreatitis is a kind of acute pancreatitis caused by the abnormal high serum triglyceride; due to the disorder of lipid metabolism, it is often combined with other endocrine metabolic disorders [44]. Hitherto, the pathogenesis of hypertriglyceridemic pancreatitis is not very unclear; however, it is clear that high concentration of TG in serum can activate pancreatic lipase and produce a large amount of free fatty acids which may damage the capillaries and cell membrane of the pancreas; this process may release cytokines and inflammatory mediators, which can lead to pancreatitis [3]. With its acute onset, severe illness, high incidence of complications, and poor prognosis, hypertriglyceridemic pancreatitis is often complicated with systemic inflammatory response syndrome (SIRS) and even multiple organ dysfunction syndrome (MODS) in the early stage [45–47]. In this study, hypertriglyceridemic AP accounted for the highest proportion in SAP, and BISAP, Ranson, APACHE-II, and MCTSI scores were significantly higher in hypertriglyceridemic AP than the other two groups, which indicated that hypertriglyceridemic AP was serious and complex in clinical practice. In terms of complications, both of the early local and systemic complications of hypertriglyceridemic AP were significantly higher than those of acute biliary AP and alcoholic AP, and the mortality rate was significantly higher than the other two groups; the difference was statistically significant. Several clinical researches [3, 48–50] indicated that from the comparison of severity and complications between different types of AP, hypertriglyceridemic AP had higher rate of complication incidences and mortality than other types of AP; this was highly in coincidence with the results of our study, and it was worth noting that with the increasing number of hypertriglyceridemia patients, the incidence of hypertriglyceridemic AP is rising, and age of onset is becoming younger and younger increasingly [51]. In some areas of China, the incidence rate of hypertriglyceridemic AP even exceeds alcoholic AP and had become the second type of AP next to the ABP [52].

## 5. Conclusions

In conclusion, the difference in etiology had obvious influence on the complications and prognosis of AP patients. The incidence rate of hypertriglyceridemic AP is increasing and becoming younger and its local and systemic complications and mortality are significantly higher than those of other types of acute pancreatitis. The presented study still have room for improvement, the risk factors for different type of AP need to be further investigate, and proper advise for the invention and treatment of AP can be put up with. Therefore, a comprehensive investigation of the pathogenesis and management of AP is needed. Meanwhile, the high-fat diet control, aerobic exercise recommendation, and early intervention of hyperlipidemia have important implication for preventing hypertriglyceridemic AP.

## Figures and Tables

**Figure 1:** Comparison of clinical classification of three groups of AP patients. (a) Mild acute pancreatitis patients; (b) moderately severe acute pancreatitis patients; (c) severe acute pancreatitis patients; there was no significant difference between groups with the same letters and hand significant difference between the groups with different letters. *p* for trend: Cuzick trend chi-square test (multiple groups).

**Figure 2:** Comparison of severity score of three groups of AP patients. (a) BISAP score of three groups; (b) Ranson score of three groups; (c) APACHE-II score of three groups; (d) MCTSI score of three groups; there was no significant difference between groups with the same letters and hand significant difference between the groups with different letters.

**Figure 3:** Comparison of local complications between three groups of AP patients in early stage. (a) The incidence rate of APFC in three groups; (b) the incidence rate of ANC in three groups; (c) the incidence rate of PPC in three groups; (d): the incidence rate of WON in three groups; (e) the incidence rate of IPN in three groups; there was no significant difference between groups with the same letters and hand significant difference between the groups with different letters. *p* for trend: Cuzick trend chi-square test (multiple groups).

**Figure 4:** Comparison of systemic complications and mortality between three groups of AP patients in early stage. (a) The incidence rate of SIRS in three groups; (b) the incidence rate of OF in three groups; (c) the incidence rate of sepsis in three groups; (d) the incidence rate of IAH in three groups; (e) the mortality rate in three groups; there was no significant difference between groups with the same letters and hand significant difference between the groups with different letters. *p* for trend: Cuzick trend chi-square test (multiple groups).

**Table 1:** Basic clinical data of three groups of AP patients.

Typing of AP	Group I (*n* = 520)	Group II (*n* = 69)	Group III (*n* = 198)	*p* value
Sex (male/female)	141/379 (27.1/72.9)	67/2 (97.1/2.9)	162/36 (81.8/18.2)	<0.01^Ф^
Age	65.0 ± 3.4	46.0 ± 2.8	38.0 ± 2.4	<0.01^Ф^
Pulse rate at admission (time/min)	92.0 ± 3.5	101.0 ± 3.2	126.0 ± 4.2	<0.01^Ф^
Respiratory rate at admission (time/min)	17.0 ± 1.2	19.0 ± 1.5	25.0 ± 1.4	<0.01^§^
WBC (×10^9^/L)	12.3 ± 1.5	14.4 ± 1.4	15.8 ± 1.2	0.167
CRP (mg/L)	45.0 ± 12.3	68.0 ± 16.7	123.0 ± 24.2	<0.01
Serum creatinine (*μ*mol/L)	62.0 ± 7.8	65.0 ± 8.2	125.0 ± 19.8	<0.01^§^
BNN (mmol/L)	5.4 ± 0.5	6.7 ± 0.7	27 ± 2.5	<0.01^§^
Blood glucose (mmol/L)	6.3 ± 0.4	7.1 ± 0.5	14.5 ± 2.0	<0.01^§^
Serum amylase (U/L)	987.0 ± 23.1	1023.0 ± 45.3	1110.0 ± 68.2	0.231
Serum calcium (mmol/L)	2.6 ± 0.3	2.4 ± 0.4	1.9 ± 0.2	0.472
Arterial pH	7.4 ± 0.2	7.4 ± 0.1	7.3 ± 0.3	0.564
Serum triacylglycerol (mmol/L)	1.7 ± 0.3	2.2 ± 0.5	21.4 ± 5.5	<0.01^§^

Group I: acute biliary pancreatitis; group II: acute alcoholic pancreatitis; group III: hypertriglyceridemic pancreatitis; WBC: White blood cell; CRP: C-reactive protein; BUN: blood urea nitrogen. ^Ф^*p* < 0.01: the difference between any two groups was statistically significant. ^§^*p* < 0.01: the difference between group III and group I or group II was statistically significant.

**Table 2:** Results of clinical classification and severity score of three groups of AP patients.

Typing of AP	Group I (*n* = 520)	Group II (*n* = 69)	Group III (*n* = 198)	*p* value
Clinical classification				
MAP	413 (79.4)	21 (30.4)	21 (10.6)	<0.01^Ф^
MSAP	75 (14.4)	25 (36.2)	53 (26.8)	<0.01^Ф^
SAP	32 (6.2)	23 (33.4)	124 (62.6)	<0.01^Ф^
BISAP score ($\bar{x}\pm s$, d)	2.1 ± 0.8	2.4 ± 1.3	4.5 ± 1.2	<0.01^§^
Ranson score ($\bar{x}\pm s$, d)	2.5 ± 0.3	2.8 ± 0.1	5.9 ± 0.4	<0.01^§^
APACHE-II score ($\bar{x}\pm s$, d)	8.4 ± 1.6	15.2 ± 2.3	20.12 ± 3.1	<0.01^Ф^
MCTSI score ($\bar{x}\pm s$, d)	3.5 ± 0.8	6.4 ± 1.1	9.2 ± 1.3	<0.01^Ф^

Group I: acute biliary pancreatitis; group II: acute alcoholic pancreatitis; group III: hypertriglyceridemic pancreatitis; MAP: mild acute pancreatitis; MSAP: moderately severe acute pancreatitis; SAP: severe acute pancreatitis; APACHE-II: acute physiology and chronic health evaluation; MCTSI: modified computed tomography severity index. ^Ф^*p* < 0.01: the difference between any two groups was statistically significant. ^§^*p* < 0.01: the difference between group III and group I or group II was statistically significant.

## Data Availability

The simulation experiment data used to support the findings of this study are available from the corresponding author upon request.
